# Clinical Analysis of Color Doppler Ultrasound Diagnosis of Senile Cataract Based on Intelligent Processor

**DOI:** 10.1155/2022/1037439

**Published:** 2022-04-27

**Authors:** Yanyan Chen, Xuebing Xiao, Lan Wu, Yang Liu

**Affiliations:** Daqing Oilfield General Hospital, Daqing 163001, China

## Abstract

In order to improve the effect of on-the-spot diagnosis of senile cataract, this paper combines the intelligent processor to explore the application of color Doppler ultrasound in the clinical analysis of senile cataract. Moreover, this paper measures and calculates the diameter, perimeter, area, volume, or velocity of blood flow reflected by color Doppler ultrasound images. In addition, this paper adopts the measurement method provided by composite measurement to design the intelligent processor. Each measurement analysis package is defined as an independent class, and the data, properties, and methods are encapsulated in a class, which is beneficial to the modular design of the program and the overall management of the system. The experimental results verify that the intelligent processor proposed in this paper has a certain effect in the clinical analysis of color Doppler ultrasound diagnosis of senile cataract.

## 1. Introduction

Cataract is currently the number one blinding eye disease in the world, and its total number accounts for half of the world's blindness [1]. The most common one is age-related cataract, and aging is a key factor in the formation of senile cataracts. Cataracts lose the normal transparency of the human lens, and the lens mainly contains protein and water. When the protein aggregates together, it will form opacity, resulting in a decrease in the transparency of the lens and the formation of cataracts [2]. At present, there are three main types of opacity in senile cataract, including cortical opacity, nuclear opacity, and posterior subcapsular opacity. Since there is a relationship between the classification of senile cataract and some clinical diseases, we can conduct statistical analysis to find the correlation, and objective data support will lead to an objective result and conclusion. For example, for people with high myopia, we can discuss the types of cataracts they focus on, look for the relationship between them, and even find out the possible causes of cataracts in people with high myopia [3].

In addition to the physical damage caused by vision loss, the decline of quality of life in elderly cataract patients may have a greater impact on quality of life. The visual acuity of senile cataract patients gradually declines, and the function of various organ systems degenerates and weakens during the aging process. Therefore, patients reduce going out, withdraw from social activities, change social roles, and reduce self-care ability, interpersonal sensitivity, and social adaptability. Moreover, visual impairment makes senile cataract patients prone to different psychological reactions from healthy people, such as anxiety, low self-esteem, low self-efficacy, and other different psychological disorders. The visual impairment caused by cataract has seriously affected the quality of life of elderly patients. Among them, the common mental health problem of senile cataract patients is the low level of self-esteem. In recent years, some studies have tried to explore their psychological problems and their care, focusing on how to improve the self-esteem and self-efficacy of the elderly and improve their quality of life. The self-esteem level of the elderly is related to gender and education level. The self-esteem level of men in early old age is higher than that of women, and the self-esteem level of women and the elderly with higher education level is relatively higher in late old age.

With the sharp rise in the elderly population, the prevalence of senile cataract is high. Most of the research on its health management and daily care is about health status, self-efficacy, and quality of life, and the psychological problems such as self-esteem caused by the health status of senile cataract patients, as well as the impact on quality of life, have begun to attract academic attention. Therefore, there is a need for mental health research on senile cataract patients and to understand their specific conditions. In-depth analysis of the relationship between the level of self-esteem and self-efficacy and their quality of life in patients with senile cataract will provide a theoretical basis for the implementation of targeted nursing interventions and the formulation of health management policies for the elderly in the future, so as to effectively improve their quality of life.

This paper combines the intelligent processor to explore the application of Color Doppler ultrasound in the clinical analysis of senile cataract, improve the clinical diagnosis effect of senile cataract, and provide a good foundation for the subsequent diagnosis and treatment of senile cataract.

## 2. Related Work

The biggest risk factor for cataracts in humans is age. The vast majority of cataracts occur in the elderly. Many drugs can induce cataracts in experimental animals. Therefore, it is unclear whether the pathway that causes lens opacity in experimental animals is similar to that in humans [4]. A common cause of visual impairment in the elderly is age-related cataracts, which are classified as nuclear, cortical, or posterior subcapsular, accounting for 29.7%, 22.9%, and 8.4% of the three types, respectively [5]. Each of these three different forms of cataract has its own set of multifactorial epidemiology, all involving multiple environmental and genetic risk factors. The genetic risk of hereditary congenital cataracts involves fewer gene or locus variants than senile cataracts, and age-related cataracts may be due to their complex inheritance patterns and late onset, making related research more difficult [6]. Age-related cataract (ARC) is influenced by genetic factors, and the genetic sequence variation of age-related cataract increases the background risk of the disease and the risk of individual exposure to the environment, so that under the influence of environmental factors accumulated over several years, individuals who have mutated are more susceptible to external factors [7]. Cataract is a multifactorial disease. In addition to genetic factors, the incidence and development are also related to factors such as age, gender, ultraviolet radiation, radiation, oxidation, physical damage, nutrition, and medication, which can lead to abnormal gene expression and affect the lens and transparency, eventually forming cataracts [8].

Cataract is a complex disease that gradually appears with aging. It may be the result of the combined action of the environment (such as sunlight and smoking) and the pathogenic gene. There are different opinions about the pathogenic gene of cataract, a genetic disease. The vast majority of cataracts are caused by the spontaneous breakdown of human long-lasting macromolecular proteins in the lens. The breakdown of long-lasting proteins is the most important of these, and recent proteomic analyses have enabled the identification of specific lens proteins and precise sites of amino acid modifications. Analysis of cataractous lens proteins has shown that sites on certain structural proteins consistently exhibit higher levels of damage than age-appropriate lenses. For age-related cataracts, nuclear opacities are predicted to be genetic in 35 to 48 percent and cortical opacities in 24 to 58 percent [9]. Of course, there are also some who carry underlying genetic factors but do not show it. The online Mendelian Inheritance in Human database claims at least 42 loci identified as isolated hereditary or primary cataract. Of the 12 mutations in crystallins, there are 100 different mutations in 100 different families. The identified mutations reported to date account for 40 to 50 percent of all autosomal dominant cataracts [10]. In addition to genetic mutations, transmembrane transport-related proteins and membrane-related proteins have a variety of functions, and they are related to the transport of various substances, protein cross-linking, or enzyme function, so changes in these proteins are also related to cataracts. There is a certain relationship between the genetics of the lens cytoskeleton; the genes encoding the lens cytoskeleton or the genes encoding the effective components in the protein directly affect the function of the cytoskeleton, which is also a kind of genetic factor [11]. Mutations in transcription factors involved in eye development can also lead to cataracts. In addition to polygenic inheritance and metabolic disorders that may be associated with cataracts, at least 42 genes and loci have been found to underlie the occurrence of isolated or primary hereditary cataracts. These pathogenic genes can be roughly divided into two categories. The first category is related to the main structure of the lens, such as *α*-protein, *β*-protein and *γ*-protein (such as CRYAA, CRYBB2, CRYGD, etc.), and *α*-catenin (GJA3, GJA8, etc.), or some other abundant membrane/cytoskeleton-related proteins (such as MIP/AQP0 and BFSP2). The second category is mainly related to the developmental process or regulatory pathway of the lens, which includes some transcription factors (such as HSF4 and PITX3), and an extended cohort of multifunctional genes (such as EPHA2, TDRD7, and FYCO1) [12].

Given the complexity of the nutritional structure in human society, it will be more elusive than we think when looking for the relationship between the intake and lack of a particular nutrient and the relationship between different diets and the risk of age-related cataract development. Because the differences between different individuals will affect the absorption of nutrients, the social economy and regional culture have created differences in the dietary structure of individuals, and some may use dietary supplements for a long time. Coming out has become a huge challenge [13]. We can currently assume that nutritional factors play an important role in the pathogenesis of cataracts, but researchers do not fully understand it. In addition, in the pathogenesis of uveitis, the microbes in the intestinal tract play a role in the pathological process [14]. Whether this role is also related to the occurrence of cataract, there is no relevant research at present.

Studies have shown that for some common causes of death (accidents, cardiovascular and cerebrovascular diseases, cancer, infectious diseases, lung diseases, etc.), the mortality rate of men is higher than that of women [15]. Blindness and moderate to severe visual impairment are more prevalent in women than in men (adjusted for age) in all regions of the world. The proportion of blind and visually impaired people varies greatly in different parts of the world. For persons older than 50 years, the prevalence of blindness and moderate to severe visual impairment is 4-6% in Africa and 16-24% in Asia [16].

## 3. Design of Intelligent Processor for Color Doppler Ultrasound Diagnosis

The basic measurement function is one of the necessary functions of ultrasonic diagnostic equipment, which is to measure and calculate the diameter, perimeter, area, volume, or blood flow velocity of the eyeball reflected in the ultrasonic image. Sonographers can detect, analyze, and diagnose diseases based on whether the measurements are within normal ranges. Therefore, the principles that must be followed when writing measurement function modules are as follows:

1. The measurement results are accurate
2. It is easy to operate and provides users with a reasonable and friendly human-computer interaction method to improve work efficiency

The basic measurement contents that can be performed by the intelligent processor are as follows, as shown in Table 1.

The main control program receives the basic measurement events on the operation control panel, loads the basic measurement filter component, and sets the basic measurement item list (for switching) according to the currently available mode. It displays measurement items according to the currently active mode and sets shared variable values required for basic measurement. Then, it waits to receive keyboard F1-F5 keys. If there is such a key, it selects the corresponding measurement item from the basic measurement callback array, loads the basic measurement dynamic library, and starts the measurement. During the measurement process, when the mouse moves, a CallBack message is sent to the display control dynamic library, and the display control dynamic library receives the message for display and sends a custom callback message to the master. The main control program receives the message, calls into the measurement function currently being executed by the basic measurement dynamic link library, and judges whether to execute the next stage according to the parameters in the message. In this way, a large cycle is established between the main control program, the basic measurement dynamic library, and the display control dynamic library. The measurement stage, display state, and callback control are well combined and coordinated to complete the basic measurement, as shown in Figure 1.

### 3.1. Console Control Event

The hardware designer writes a special keyboard control program for SKY-800, receives each key on the console, and outputs the specified code. The home-made keyboard control component receives the code and binds the corresponding events. The main control program controls the system by responding to events.

### 3.2. Keyboard Filtering

All keys on the control panel should not work at all times. For example, in the mode B control, the PRF, Steer, and other keys should not be able to perform operations, and the mode cannot be switched in the measurement state. In order to solve this problem, the keyboard filter component is self-made, and different control states are loaded with different filter controls. The purpose of controlling whether each key of the keyboard is available can be achieved by loading and popping the component.

### 3.3. Measurement Display

The points, lines, ellipses, trajectories, and measurement results displayed on the screen during the measurement process are all sent to the Overlay control layer through the main control program, and the display and output are realized by the Overlay control layer.

### 3.4. Loading of Dynamic Link Library

Because the basic measurement dynamic library has many output functions and the interaction between the main control program and the dynamic library is frequent, the system chooses the method of statically loading the dynamic library.

### 3.5. Shared Data

The calculation of the basic measurement requires the current image information, so the image information needs to be shared between the main control program and the basic measurement dynamic link library. In addition, the current state of the measurement process is distinguished by the measurement phase. Since both the main control program and the basic measurement dynamic library program need to modify the stage value, in order to achieve the synchronization of the modification and use of the stage value, the measured stage variables must be shared.

### 3.6. Multilanguage Switching

The multilanguage display of the basic measurement results is realized through the callback function. The multilanguage module in the main control program defines the multilanguage execution function and function body. The basic measurement dynamic library remotely calls back the multilanguage functions in the main control program to complete the multilanguage switch. In this way, code duplication is avoided, and it is beneficial to the modification of the program and the unification of the output.

Image information must be obtained for measurement calculations. When switching modes and modifying parameters, the content in the image information structure is modified to ensure accurate measurement results.

#### 3.6.1. B Mode Measurement

The image presented by the B mode is a two-dimensional grayscale image of a cross-section inside the eyeball or tissue. Therefore, it is possible to measure the distance, perimeter, and area of eyeball cross-section through image display. The volume of the eyeball can be calculated based on the measurement of the distance between the cross-section and the longitudinal section of the eyeball.

*(1) The Straight Line Method Measure Distance*. In the measurement method, it gives the start and end points of the distance to be measured, *P*_*s*_ and *P*_*e*_.

The following is the measurement formula:

(1) $$\begin{array}{c} D=\frac{\sqrt{{\left(P_{c}x-P_{s}\cdot x\right)}^{2}+{\left(P_{e}\cdot y-P_{s}\cdot y\right)}^{2}}}{\text{BDotPerMm}}. \end{array}$$

*(2) The Ellipse Method Measures the Five Perimeter and Area*. In the measurement method, it gives the major and minor axes of the ellipse, *P*_*s*_, *P*_*e*_, and *r*.

The following is the measurement formula:

(2) $$\begin{array}{c} C=\frac{\pi \cdot \sqrt{2\cdot \left[\left(\left({\left(P_{e}\cdot x-P_{s}x\right)}^{2}+{\left(P_{e}\cdot y-P_{s}\cdot y\right)}^{2}\right)/4\right)+r^{2}\right]}}{\text{BDotPerMm}},\\ A=\frac{\pi \cdot \left(\left(\sqrt{{\left(P_{e}.x-P_{s}.x\right)}^{2}+{\left(P_{e}.y-P_{s}.y\right)}^{2}}\right)/2\right)\cdot r}{{\text{BDotPerMm}}^{2}}. \end{array}$$

*(3) The Trajectory Method Measures the Perimeter and Area*. In the measurement method, according to the range to be measured, it circles the boundary by itself.

The following is the measurement formula:

(3) $$\begin{array}{c} C=\overset{\text{Num}}{\underset{i=0}{\sum }}\frac{D_{i}}{\text{DotPMm}},\;\text{C Num is the number of points on the track},\\ A=\text{Double integral formula}\approx \sum \frac{X_{1}*Y_{2}-X_{2}*Y_{1}}{{\text{DotPMm}}^{2}}. \end{array}$$

*(4) Three Straight Lines to Measure the Volume*. In the measurement method, the length and height are marked with straight lines on the cross section (or longitudinal section) of the eyeball to be measured, and then, the thickness is marked with straight lines on the longitudinal section (or cross-section).

The following is the measurement formula: *D*_1_, *D*_2_, *D*_3_ is three distance values.

(4) $$\begin{array}{c} V=\frac{\pi *D_{1}*D_{2}*D_{3}}{6}. \end{array}$$

#### 3.6.2. M Mode Measurement

The ultrasound image of the M mode shows the movement of the inner eyeball organ, which is especially suitable for the inspection of the eyeball. The image formation of the M mode is to expand the position of the received echo in time to form a trajectory map of the movement of each point in one-dimensional space in time, so the image of the M mode is a depth-time map. That is, the horizontal axis is the slow scan time, and the vertical axis is the fast scan depth position.

*(1) Distance Measurement*. The measurement method is basically the same as the measurement of the B mode distance, except that the M mode distance measurement should be perpendicular to the horizontal axis, because the M mode is a one-dimensional map. Only distances at the same time are meaningful to study.

*(2) Eye Movement Frequency*. In the measurement method, it marks an eye movement cycle with start and end points.

In the measurement formula, *D* is the distance between the eye movement cycles on the image.

(5) $$\begin{array}{c} \text{HR}=\frac{60*\text{MDotPSec}*\text{MDotPMm}}{D}. \end{array}$$

#### 3.6.3. D Mode Measurement

D mode ultrasound image shows the blood flow spectrum of blood vessels. The image is a velocity-time graph, the abscissa represents the duration of blood flow, the ordinate represents the magnitude of blood flow velocity, and the horizontal line in the spectrogram is the baseline. The frequency-shifted signal above the baseline is positive and represents blood flow towards the probe. The frequency-shifted signal below the baseline is negative, representing blood flow away from the probe. In addition, the spectral gray scale represents the relative number of red blood cells that have the same flow rate within the sampling volume. The greater the number of blood cells, the darker the grayscale, otherwise, the lighter the grayscale.

*(1) Peak Speed*. In the measurement method, it marks the position of the systolic or diastolic peak in the eye movement cycle with dots.

In the measurement formula, BaseLINE is the baseline position, *θ* is the sampling angle, and Invert is the axis inversion.

(6) $$\begin{array}{c} \text{Vel}=\frac{\left(Y-\text{BaseLine}\right)\times \text{Invert}\times \text{Cos}\theta }{\text{ DotPVel }},\\ \text{Time}=\frac{\text{ Dot }}{\text{ DDotPSec }}\;\left(\text{Dot is the distance between two peaks}\right),\\ \text{Acc}=\frac{{\text{Vel}}_{A}-{\text{Vel}}_{B}}{\text{ Tim}{\text{e}}_{A}-\text{Tim}{\text{e}}_{B}}. \end{array}$$

*(2) Two-Peak Speed Ratio*. In the measurement method, it marks the position of the two peak points to be compared with dots.

In the measurement formula, Vel_*A*_ and Vel_*B*_ are two peaks, respectively.

(7) $$\begin{array}{c} \frac{A}{B}\%=\frac{{\text{Vel}}_{A}}{{\text{Vel}}_{B}}*100\%. \end{array}$$

The composite measurement analysis module provided by the intelligent processor ultrasound diagnosis system includes multiple analysis packages. Composite measurement is to summarize the measurement reference items commonly used by clinicians and then categorize them into different measurement software packages. The analysis results are displayed on the screen, and the composite measurement results can also be automatically loaded into the report, and the report provides preview and print output functions to facilitate the user's diagnosis, use, and output.

The measurement method and design structure provided by the composite measurement are basically the same as the basic measurement. The composite measurement design method fully embodies the concept of class in object-oriented programming. Moreover, each measurement analysis package is defined as an independent class, and the data, properties, and methods are encapsulated in a class, which is beneficial to the modular design of the program and the overall management of the system. The design ideas of each composite measurement analysis package are basically the same.

When the main control program and the overlay control layer control the composite measurement, the structures pointed to by the IParam parameter pointer in the transmission message are, respectively, the structures transmitted by the main control program to the Overlay control layer, as shown in Table 2, and the structures returned by the Overlay control layer to the main control layer, as shown in Table 3.

## 4. Clinical Analysis of Color Doppler Ultrasound Diagnosis of Senile Cataract Based on Intelligent Processor

Combined with the intelligent processor designed in the third part, this paper conducts a clinical analysis on the effect of color Doppler ultrasound in diagnosing senile cataract. In this paper, the data of cataract patients in the hospital outpatient department in the coming year are collected as research samples, the content is shown in Figure 2. The patient was placed in the supine position, and the double eyelid was gently closed and the couplant is applied. At the same time, it is necessary to instruct the patient to rotate the eyeball to fully display the lens structure, observe and measure the thickness of the lens, axial length, etc. in turn, observe the echo of the lens capsule, the sound transmission of the lens and vitreous, and the sonographic changes of the retina, choroid, eyeball wall and other intraocular structures. When checking, we first use two-dimensional real-time scanning and, if necessary, add color flow imaging, and try to reduce the pulse repetition frequency and wall filtering until no noise artifacts appear. The pulse Doppler angle is <15°.

In this paper, a statistical study was conducted through multiple groups of experiments to explore the comparison of the data of normal peers and senile cataract patients. Moreover, this paper separately counts peak systolic blood flow velocity (PSV), end-diastolic blood flow velocity (EDV), average blood flow velocity (TAMX), and resistance index (RI). The statistical results are shown in Tables 4–7.

## 5. Analysis and Discussion

The destruction of the lens capsule caused by various factors or the increase of its permeability and the loss of its barrier function or the disorder of lens metabolism and the degeneration of the main component of crystallin, the appearance of small fissures, vacuoles, and epithelial cell proliferation among the fibers make the transparent lens cloudy, which can be called cataract. Senile cataract is one of the most common acquired primary cataracts, and the older the age, the higher the incidence. Lens opacities in most cataract patients start from the periphery, and the visual impact is not obvious. Moreover, they have no special discomfort, and it is difficult to attract attention, so that when they develop to affect their vision, they come to the hospital and miss the opportunity of drug treatment. When it develops to maturity, the surgeon cannot directly observe the condition of the fundus. In particular, vitreous lesions, fundus lesions, retinal detachment, and retrobulbar space-occupying lesions may be masked by cataracts in advanced senile cataract patients. Therefore, preoperative ultrasonography for senile cataract patients has the following significance: (1) It can understand whether there are lesions in the vitreous body, retina, and retrobulbar of the patient and guide the surgeon to choose the correct and appropriate surgical method. (2) It can accurately detect the opacity of the lens, measure the diameter of the eye and whether other lesions are combined in the eye, and create conditions for clinical grasping and striving for good surgical opportunities. (3) The measurement of the eye axis can provide a reliable basis for calculating the refraction of intraocular lens during surgery. (4) The detection of comorbidities can provide objective basis for surgical plan and prognosis. (5) The visual effect after cataract surgery is good, but some patients have high vision expectations regardless of their own eye conditions. The transparency of the vitreous body and the presence or absence of retinal detachment play a decisive role in the recovery of visual acuity after cataract surgery. Preoperative ultrasonography has a relatively objective basis for the evaluation of patients' vision and prognosis. It will provide a convincing objective basis when doing ideological work for these patients and can also avoid unnecessary disputes after surgery.

The above research verifies that the intelligent processor proposed in this paper has a certain effect in the clinical analysis method of color Doppler ultrasound diagnosis of senile cataract.

## Figures and Tables

**Figure 1:** Workflow of the basic measurement module.

**Figure 2:** Some sample images.

**Table 1:** Basic measurement content.

Operating mode	Measurement item	Measurement methods
B mode	Distance	Straight line method
	Perimeter	Ellipse and trajectory method
	Area	Ellipse and trajectory method
	Volume	Three distances, ellipse+distance
M mode	Distance	Straight line method
	Eye movement frequency	Two-point method
D mode	Peak speed	Two-point method, trajectory method
	A/B	Two-point method

**Table 2:** The structure of the master transmission.

Name	Instruction
MeasReg	Measurement area
BeginPoint	Measurement or text display start position
CursorType	Cursor display type
Text	Output text
PointArray	Coordinate values of all points of the track
PointNum	The number of all points of the track

**Table 3:** Structures returned by the overlay control layer.

Name	Instruction
PoimY	Point ordinate
Radius	Ellipse minor axis
Startp	Line start point coordinates
EndP	Line end point coordinates
PointArray	Coordinate values of all points of the track
PoimCouat	The number of all points of the track

**Table 4:** Comparison of PSV between normal healthy people of the same age and senile cataract patients (xm/s).

Number	Healthy group	Cataract group	Number	Healthy group	Cataract group
1	13.76	8.33	19	13.07	10.47
2	12.78	9.94	20	13.02	9.16
3	8.87	9.68	21	9.37	9.25
4	10.57	10.46	22	9.73	10.55
5	13.08	10.91	23	8.54	10.17
6	12.47	8.43	24	9.53	7.80
7	8.64	8.98	25	9.04	7.96
8	11.07	8.30	26	8.60	10.13
9	11.74	8.05	27	11.54	8.60
10	10.56	10.90	28	9.06	8.23
11	8.15	9.07	29	11.45	9.04
12	12.53	9.99	30	11.06	10.89
13	12.28	10.68	31	10.64	10.68
14	12.40	9.91	32	12.80	8.15
15	11.54	9.70	33	8.29	10.93
16	10.00	10.76	34	9.65	9.26
17	13.57	10.01	35	13.72	9.78
18	8.31	7.76	36	10.66	8.75

**Table 5:** Comparison of EDV between healthy people of the same age and senile cataract patients (xm/s).

Number	Healthy group	Cataract group	Number	Healthy group	Cataract group
1	2.66	3.11	19	3.63	3.53
2	4.28	2.62	20	2.40	2.25
3	3.00	2.70	21	2.48	3.24
4	2.67	2.75	22	3.11	2.47
5	2.39	3.15	23	3.35	2.74
6	2.96	3.64	24	3.90	3.24
7	3.65	3.23	25	3.40	3.30
8	2.32	3.74	26	2.34	3.05
9	3.99	2.44	27	2.40	2.14
10	2.23	2.82	28	3.47	3.42
11	3.04	2.68	29	4.21	2.58
12	2.62	2.30	30	2.65	2.78
13	2.96	3.08	31	3.44	3.68
14	4.11	2.35	32	2.83	3.24
15	2.91	2.28	33	2.88	3.64
16	3.64	2.50	34	3.69	3.16
17	4.19	3.42	35	3.96	3.12
18	3.55	3.80	36	3.11	2.54

**Table 6:** Comparison of TAMX between normal healthy people of the same age and senile cataract patients (xm/s).

Number	Healthy group	Cataract group	Number	Healthy group	Cataract group
1	4.42	3.02	19	4.82	5.36
2	4.07	3.65	20	6.15	4.98
3	6.28	4.93	21	4.54	3.46
4	4.19	4.71	22	6.79	4.46
5	4.57	2.56	23	5.87	3.71
6	7.39	5.73	24	5.31	2.65
7	4.13	2.23	25	6.91	2.64
8	5.17	3.80	26	3.66	5.75
9	6.19	2.31	27	3.89	2.82
10	4.99	3.11	28	7.10	5.11
11	5.60	4.48	29	4.93	2.23
12	5.89	2.25	30	4.77	3.66
13	6.31	5.24	31	4.64	2.82
14	3.87	2.99	32	4.74	2.56
15	5.50	3.05	33	5.88	2.53
16	3.72	5.50	34	7.11	3.43
17	5.13	3.28	35	4.99	5.61
18	4.14	5.06	36	5.76	5.59

**Table 7:** Comparison of RI between normal healthy people of the same age and senile cataract patients (xm/s).

Number	Healthy group	Cataract group	Number	Healthy group	Cataract group
1	0.64	0.70	19	0.63	0.69
2	0.59	0.66	20	0.56	0.75
3	0.59	0.79	21	0.61	0.64
4	0.61	0.64	22	0.65	0.69
5	0.62	0.68	23	0.65	0.69
6	0.66	0.77	24	0.67	0.69
7	0.68	0.71	25	0.61	0.64
8	0.65	0.81	26	0.55	0.77
9	0.61	0.79	27	0.58	0.73
10	0.55	0.65	28	0.60	0.66
11	0.66	0.73	29	0.58	0.67
12	0.57	0.71	30	0.61	0.68
13	0.64	0.68	31	0.62	0.76
14	0.70	0.68	32	0.61	0.65
15	0.70	0.69	33	0.61	0.79
16	0.64	0.79	34	0.61	0.66
17	0.61	0.81	35	0.68	0.75
18	0.68	0.65	36	0.67	0.66

## Data Availability

The labeled dataset used to support the findings of this study is available from the corresponding author upon request.
